The article "Celecoxib Reverse Invasion and Metastasis of Gastric Cancer through Lnc_AC006548.28-miR-223-LAMC2 Pathway" was retracted in 2023. Reasons: signs of a paper mill; suspected computer-generated content; unreliable results or conclusions; concerns about the data.

# Celecoxib Reverse Invasion and Metastasis of Gastric Cancer through Lnc_AC006548.28-miR-223-LAMC2 Pathway

**DOI:** 10.1155/2022/6140727

**Published:** 2022-05-27

**Authors:** Guohua Jin, Jianguang Zhang, Tingting Cao, He Zhu, Yang Shi

**Affiliations:** Department of Gastroenterology, The First Hospital of Jilin University, Changchun, China

## Abstract

Celecoxib, a specific cyclooxygenase-2 (COX-2) inhibitor, is a traditional nonsteroidal antipyretic analgesic and anti-inflammatory drug commonly used in clinic, which has inhibitory effect on colorectal cancer, gastric cancer, and other malignant tumors. This study showed that Celecoxib could significantly reverse the invasion and metastasis of gastric cancer and improved the pathological changes due to GC. We collected the clinical specimens to analyze the correlation between the expression of Lnc_AC006548.28, miR-223, and LAMC2. In the mouse model, Celecoxib can slowdown the growth of GC tumor and the occurrence of this effect may depend on Lnc_AC006548.28-miR-223-LAMC2 pathway, in vitro transfection, RT-PCR, western blot, CCK8, small chamber assay, flow cytometry, and immunohistochemistry to retest the protective effect of celecoxib. Our results showed that Celecoxib could reverse invasion and metastasis of gastric cancer through Lnc_AC006548.28-miR-223-LAMC2 pathway.

## 1. Introduction

Gastric cancer (GC) is one of the most common malignant tumors in the world. China is a high incidence area of gastric cancer, with about 400000 new cases each year, accounting for the world's total 42% of the total cases. The 5-year survival rate of patients with early gastric cancer can reach more than 90%. However, most patients have tumor metastasis when they go to the hospital, so surgery cannot cure gastric cancer cure once and for all, and the 5-year survival rate is quite low. In recent years, with the new generation of chemotherapy drugs used in clinical, the treatment effect of advanced gastric cancer has improved, but the long-term effect is not satisfactory.

Adhesion signal plays an important role in tumor microenvironment, which can promote the development, invasion, and metastasis of cancer. Laminin-5, expressed in many epithelial tissues and tumor microenvironment, is proved to accelerate cell adhesion and metastasis [1]. LAMC2 is a member of laminin-5. It also shows that LAMC2 is associated with metastasis, recurrence, and poor prognosis of cancer [2, 3]. Studies have found that LAMC2 expression is significantly upregulated in lung adenocarcinoma metastatic cells, and high expression of LAMC2 can increase the metastasis and invasion of lung adenocarcinoma cells through epithelial mesenchymal transition (EMT), while knockdown of LAMC2 expression can reduce the metastasis and invasion of lung adenocarcinoma cells [4]. Nguyen et al. [5] found that the expression of LAMC2 was significantly upregulated in oral squamous cell carcinoma (OSCC), and the expression level of LAMC2 was significantly associated with the classification and invasion depth of OSCC. Huang et al. [6] found that LAMC2 was significantly correlated with disease specificity, recurrence, and overall survival rate of colorectal cancer. At the same time, high expression of lamc2 can promote the proliferation, metastasis and invasion of colorectal cancer cell line in vitro. In addition, Kinoshita et al. [7] found that silencing lamc2 can significantly inhibit the invasion and metastasis of head and neck squamous cell carcinoma.

In our previous study, we found that the expression of LAMC2 gene in gastric cancer tissue was significantly higher than that in normal tissue [8], suggesting that high expression of LAMC2 may play an important role in the occurrence of gastric cancer. Yamamoto et al. [9] found that Wnt5a indirectly regulates the invasiveness of gastric cancer cells by up regulating the expression of LAMC2, which suggests that the high expression of LAMC2 in gastric cancer may be caused by Wnt5a. Xu et al. [10] found that high expression of LAMC2 was significantly associated with metastasis and invasion of gastric cancer. However, the mechanism of LAMC2 involved in gastric carcinogenesis has not been fully elucidated. Therefore, we need to further explore the role of LAMC2 in the development of gastric cancer.

By completely or incompletely complementary binding with the 3ʹ end of the target mRNA, microRNA (miRNA) can inhibit the expression of the protein or induce the degradation of its mRNA, so as to regulate the expression of the target gene and then affect the proliferation, differentiation, and apoptosis of cells. At the same time, experiments in vitro showed that miR-223 can promote the proliferation, metastasis, and invasion of gastric cancer cells [11, 12]. However, which target gene miR-223 acts on, and how miR-223 participates in cancer invasion and metastasis through regulating target genes still need to be further explored.

Our team predicted that LAMC2 could be the target gene of miR-223 through bioinformatics. Long noncoding RNA (lncRNA) is a kind of noncoding RNA with a length of more than 200 nucleotides [13–15].

Celecoxib, a specific cyclooxygenase-2 (COX-2) inhibitor, is a traditional nonsteroidal antipyretic analgesic and anti-inflammatory drug commonly used in clinic, which has inhibitory effect on colorectal cancer, gastric cancer, and other malignant tumors [16]. Some studies have found that celecoxib can inhibit the invasion of gastric cancer by affecting the expression of E-cadherin, vascular endothelial growth factor, and COX-2, and also by interfering with NF-*κ*B signaling pathway, snail signaling pathway, and microvascular density [17, 18]. A recent study found that the efficacy of celecoxib is more significant than that of traditional treatment [19]. However, by which mechanism does celecoxib resist gastric cancer? What is the relationship between internal molecules and regulation?

Our previous study found that celecoxib may play a role in resisting gastric cancer by inhibiting LAMC2 expression, leukocyte metastasis, and focal adhesion [20]. Because Lnc_AC006548.28 may participate in the regulation of LAMC2 by miR-223 competitively as a ceRNA (competitive endogenous RNA), we speculate that celecoxib may pass through Lnc_AC006548.28 which interacts with miR-223 to regulate the expression of LAMC2 and reverse the occurrence of gastric cancer. This conclusion has not been reported.

## 2. Materials and Methods

### 2.1. Clinical Tissue Specimens

A total of 60 patients with gastric cancer at the first Hospital of Jilin University between February 2019 and March 2020 were enrolled in this study. Surgical specimens were examined and graded according to the Classification of Gastric Carcinoma. Inclusion criteria: (1) gastric cancer diagnosed by pathology; (2) the first treatment did not undergo radiotherapy and chemotherapy. Exclusion criteria: (1) patients with family history of tumor; (2) patients with chronic diseases such as heart, lung, liver, and kidney. Gastric cancer tissues were included in the cancer group, and tissue next to cancer was used as the control group. At the same time, 60 cases of healthy person in our hospital were selected into the blank group, among which there were 30 males and 30 females. The study was approved by the ethical committee of our hospital. Patients have signed the informed consent forms. The tissues taken from cancer group, control group, and blank group were divided into three parts, one part was used to make paraffin section, one part was used to extract RNA, and the other part was used to extract protein.

### 2.2. Animals

The breeder pairs of the Lnc_AC006548.28-KO and of the LAMC2-KO mice were purchased from the Beijing Weitonglihua Experimental Animal Technology Co., Ltd. and contained the genetic basis of the C57BL/6J mice. The animals were supplied with plenty of food and water and housed in standard cages in a light-controlled room at 25°C ± 1°C.

### 2.3. Drugs and Reagents

Celecoxib was purchased from Pfizer Pharmaceuticals LLC (American). GAPDH was purchased from HUABIO. Primary antibodies against LAMC2 were purchased from Affinity Biosciences, SYBR Premix ExTaq kit (TaKaRa Biotechnology, Dalian, China), TRIzol Reagent (Tiangen, China), and PrimescriptTM RT reagent Kit (TaKaRa Biotechnology, Dalian, China), respectively. PCR detection primers was designed and purchased by Guangzhou RiboBio Co., Ltd., China. oeLnc_AC006548.28, siLnc_AC006548.28, miR-223 mimic, miR-223 inhibitor, oeLAMC2, and siLAMC2 were designed and purchased by Guangzhou RiboBio Co., Ltd., China.

### 2.4. Mouse Model of Gastric Cancer

MKN-45, MGC-803, and NCI-N87 cells were cultured in vitro and passaged routinely. The cells were collected and washed with normal saline. The cell density was 22 × 1010/ml and was injected subcutaneously into the junction of neck and forelimb of nude mice. The tumorigenesis of nude mice was observed and measured. Indicators of successful modeling: there was no obvious inflammatory reaction after injection in nude mice. Tumor formation was observed at 45 days, and solid mass could be palpated by palpation. Under the light microscope, the nuclei of tumor tissue were large, oval or irregular, and arranged disorderly.

The mice were divided into five groups, including (1) control group (0.2 ml 0.9% normal saline for 56 days); (2) a Celecoxib group (0.2 ml Celecoxib (50 mg/kg·d)for 56 days); (3) a Celecoxib + Lnc_AC006548.28-KO group (0.2 ml Celecoxib for 56 days to Lnc_AC006548.28-KO mice); (4) a Celecoxib + OE-miR-223 group (0.2 ml Celecoxib for 56 days to OE-miR-223 mice); (5) a Celecoxib + LAMC2-KO group (0.2 ml Celecoxibfor 56 days to LAMC2-KO mice). Determination of tumor size, immunohistochemistry, and HE staining was according to previous protocols.

### 2.5. Quantitative Real-Time PCR (qRT-PCR)

The PCR reaction consisted of 2 × SYBRGREEN master mix, 0.2 *μ*M primer, and 1 *μ*l DNA in final volume of 10 *μ*l. The qPCR was run in triplicate with preincubation. The amplified product was detected using SYBR Green I and each run included a negative (ultrapure H_2_O) and a positive control.

### 2.6. Cell Culture and Experiments

MKN-45, MGC-803, or NCI-N87 cells were seeded in 96-well plate and were treated with different concentrations of Celecoxib (0, 10, 20, 30, 40, and 50 mg/L) for different time (24 h, 48 h, and 72 h). MTT assay, cell proliferation, migration, and invasion and also cell apoptosis were performed as per the previous protocols. The suitable cell line and celecoxib concentration were selected.

### 2.7. Western Blotting Analysis

We obtained the protein by collecting tissue homogenate or cells, decomposed it with lysis buffer for half an hour, and then put it into the centrifuge at 1.5 W·rpm at 4°C for 1/4H. Follow the manufacturer's requirements to trace the protein. Western blotting was performed according to our previous study using the same protocols.

### 2.8. Dual-Luciferase Reporter Assay

The MiR-223 untranslated region (3ʹUTR) sequences containing the potential binding sites of Lnc_AC006548.28 or the mutant binding sites were amplified, which were named miR-223-WT or miR-223-MUT. Then, the WT or MUT plasmids and Lnc_AC006548.28 or NC were co-transfected into cells using Lipofectamine 3000. After 24 h, the cells were harvested, and the Luciferase activity was measured using the Dual-Luciferase reporter assay system.

### 2.9. Statistical Analysis

All statistical data were analyzed using GraphPad Prism 5 (GraphPad Software, Inc., La Jolla, CA, USA). Comparisons between groups were performed using one-way analysis of variance (ANOVA) and followed by LSD post hoc. *P* < 0.05 was considered statistically significant.

## 3. Results

### 3.1. The Expression of LAMC2 Was Significantly Increased in Gastric Cancer

Clinical tissue samples were collected. There were 10 cases of gastric cancer tissue and 10 cases of paracancerous tissue. The expression of LAMC2 in paracancerous tissue was detected by immunohistochemistry (Figure 1(a)). The expression of LAMC2 in gastric cancer tissue was detected by immunohistochemistry (Figure 1(b)). The expression of LAMC2 protein in different tissues was detected by Western blot (Figure 2(a)). The LAMC2 positive percentage of the cancer tissue group was higher than that of paracancerous tissue (Figure 2(b)). LAMC2 protein in cancer tissue was higher than that in paracancerous tissue (Figure 2(c)).

### 3.2. There Was Correlation between the Expression of LAMC2，Lnc_AC006548.28 and miR-223 in Gastric Cancer Tissue

Quantitative PCR was used to detect the expression of LAMC2 mRNA, Lnc_AC006548.28, and miR-223 in cancer tissue and paracancerous tissue. The expression of LAMC2 mRNA in cancer tissues was higher than that in adjacent tissues. The expression of miR-223 in cancer tissues was lower than that in adjacent tissues. The expression of Lnc_AC006548.28 in cancer tissues was higher than that in adjacent tissues (Figure 2(d)). The correlation analysis between genes also showed the association of LAMC2, Lnc_AC006548.28 with miR-223 (Figure 2(e)).

### 3.3. Using Celecoxib and Interfering LAMC2, Lnc_AC006548.28, and miR-223 Genecan Affect the Pathological Progression of Gastric Tumor

Tumor bearing test in vivo showed that celecoxib and interference with lamc2, Lnc_AC006548.28, and miR-223 expression. The size of tumor was smaller (Figure 3(a)), and the growth of tumor slowed down (Figure 3(b)). The tumor infiltration was observed by HE staining, which showed that using celecoxib or KO Lnc_AC006548.28, OE-miR-223, and KO LAMC2. The area of tumor necrosis and apoptosis decreased (Figure 4(a)). The difference was statistically significant (Figure 4(c)). These results suggest that LAMC2 may regulate Lnc_AC006548.28 by regulating miR-223 expression and affect the pathological progress of tumor. Ki67 was used to detect the proliferation of cancer cells; the same results were obtained (Figures 4(b) and 4(d)).

### 3.4. Celecoxib Exerts Antitumor Effect through Lnc_AC006548.28-miR-223-LAMC2 Pathway

Suitable primers were designed (Figure 4(e)). PCR test showed that the expression of genes in different groups showed the relationship of ebb and flow, and the difference was statistically significant, suggesting that the expression of these genes had the role of mutual regulation (Figure 4(f)).

### 3.5. There was Correlation between the Expression of LAMC2, Lnc_AC006548.28, and miR-223 under Celecoxib Treatment In Vitro Cell Model

The suitable cell line and celecoxib concentration were selected for follow-up test. MKN-45 cell and 40 mg/L were chosen (Figure 5(a)). Western blot showed that the expression of LAMC2 protein was positively correlated with the expression of Lnc_AC006548.28 and negatively correlated with the expression of miR-223 (Figure 5(b)). RT-PCR results also showed that the expression of LAMC2 mRNA was positively correlated with the expression of Lnc_AC006548.28 and negatively correlated with the expression of miR-223 (Figure 5(c)).

### 3.6. Celecoxib Attenuates the Pathological Changes of MKN-45 Cells through Lnc_AC006548.28-miR-223-LAMC2 Pathway

CCK8 experiment showed that, after inhibiting the expression of LAMC2 and Lnc_AC006548.28 and enhancing the expression of miR-223, cell proliferation was decreased, and the difference was statistically significant (Figure 6(a)). Boyden chamber assay showed that, after inhibiting the expression of LAMC2 and Lnc_AC006548.28 and enhancing the expression of miR-223, cell migration and invasion ability was decreased (Figure 6(b)), and the difference was statistically significant (Figure 6(c)). Flow cytometry experiment showed that, after inhibiting the expression of LAMC2 and Lnc_AC006548.28 and enhancing the expression of miR-223, cell apoptosis was increased (Figure 7(a)), and the difference was statistically significant (Figure 7(b)). Dual-luciferase assay also proved the regulatory relationship among Lnc_AC006548.28, miR-223, and LAMC2. The difference was statistically significant (Figure 7(c)).

## 4. Discussion

The objective of this research was to find out the pharmacological effects of Celecoxib on Gastric cancer. We discussed the relationship between Lnc_AC006548.28, miR-223, and LAME2 and the pathogenesis of gastric cancer and explored the relationship and mechanism between them and the pathogenesis of gastric cancer after celecoxib. We also found Lnc_AC006548.28, miR-223, and LAMC2 are potential therapeutic targets for gastric cancer.

This study intended to explore the regulatory relationship between AC006548.28, miR-223, and LAMC2 by knockout, overexpression, and double luciferase method. At the same time, the relationship between celecoxib and the pathogenesis of gastric cancer was studied at the three levels of tissue, cell, and animal model, and the mechanism of celecoxib through Lnc_AC006548.28-miR-223-LAMC2 pathway can affect the development of gastric cancer and provide new ideas for the treatment of gastric cancer. If common and cheap celecoxib can be used to intervene the development of gastric cancer, it can greatly reduce the economic burden of patients and then reduce the social burden.

## 5. Conclusions

In conclusion, Celecoxib could reverse invasion and metastasis of gastric cancer through Lnc_AC006548.28-miR-223-LAMC2 pathway.

## Figures and Tables

**Figure 1:** LAMC2 in paracancerous and gastric cancer tissues detected by immunohistochemistry. (a) 10 cases of paracancerous tissue samples were collected; the expression of LAMC2 in paracancerous tissue was analyzed by immunohistochemistry; (b) 10 cases of gastric cancer tissue samples were collected; the expression of LAMC2 in gastric cancer tissue was detected through immunohistochemistry.

**Figure 2:** Correlation analysis between the expression of LAMC2, Lnc_AC006548.28, and miR-223 in gastric cancer tissue. (a) The protein level of LAMC2 in different tissues was detected by western blot; (b) the positive percentage of LAMC2 was detected by RT-PCR; it was higher in cancer tissue group than that of paracancerous tissue group; (c) the expression of LAMC2 protein was detected by western blot; the protein level in cancer tissue was higher than that in paracancerous tissue; (d) quantitative PCR was used to detect the expression of LAMC2 mRNA; the expression of Lnc_AC006548.28 in cancer tissues was higher than that in adjacent tissues; (e) the correlation between the expression of LAMC2, Lnc_AC006548.28 and miR-223 was detected by correlation analysis between genes.

**Figure 3:** The size of tumor in different groups. (a) The size of tumor was detected after treatment with lamc2; (b) the tumor growth rate was detected after treatment with lamc2.

**Figure 4:** Celecoxib exerts antitumor effect through Lnc_ AC006548.28-miR-223-LAMC2 pathway. (a and c) After the treatment with celecoxib or KO Lnc_AC006548.28, OE-miR-223, and KO LAMC2 detected the tumor infiltration by HE staining. The difference was statistically significant. (b and d) Ki67 was used to detect the proliferation of cancer cells; the same results were those that suggest LAMC2 may regulate Lnc_AC006548.28 by regulating miR-223 expression and affect the pathological progress of tumor. (e) Suitable primers were designed. (f) The expression of genes in different groups was detected by PCR test, the difference was statistically significant, and the expression of these genes had the role of mutual regulation.

**Figure 5:** LAMC2 was positively correlated with the expression of Lnc_AC006548.28 and negatively correlated with the expression of miR-223. (a) The suitable cell line and celecoxib concentration were selected by follow-up test. At last, MKN-45 cell and 40 mg/L were used. (b) The cells were collected; the expression of LAMC2 protein and the expression of Lnc_AC006548.28 were detected by western blot. (c) RT-PCR detected the mRNA levels the expression of LAMC2, Lnc_AC006548.28, and miR-223.

**Figure 6:** Cell proliferation, migration, and invasion detected by CCK8 and Boyden chamber assay. (a) Through inhibiting the expression of LAMC2 and Lnc_AC006548.28 and enhancing the expression of miR-223, cell proliferation was detected by CCK8 experiment; (b, c) through inhibiting the expression of LAMC2 and Lnc_AC006548.28 and enhancing the expression of miR-223, cell migration and invasion ability were detected by Boyden chamber assay. The difference was statistically significant.

**Figure 7:** Regulatory relationship among Lnc_AC006548.28, miR-223, and LAMC2. (a, b) Through inhibiting the expression of LAMC2 and Lnc_AC006548.28 and enhancing the expression of miR-223, cell apoptosis was detected by flow cytometry experiment; the difference was statistically significant. The regulatory relationship among Lnc_AC006548.28, miR-223, and LAMC2 was detected through Dual-luciferase assay. The difference was statistically significant.

## Data Availability

The datasets used and analyzed during the current study are available from the corresponding author upon reasonable request.
